The article "Electronic Nose for Differentiation and Quantification of Yeast Species in White Fresh Soft Cheese" was retracted in 2023. Reasons: signs of a paper mill; suspected computer-generated content; unreliable results or conclusions; concerns about the data.

# Electronic Nose for Differentiation and Quantification of Yeast Species in White Fresh Soft Cheese

**DOI:** 10.1155/2022/8472661

**Published:** 2022-01-17

**Authors:** Nawaf Abu-Khalaf, Wafa Masoud

**Affiliations:** Department of Agricultural Biotechnology, Faculty of Agricultural Sciences and Technology, Palestine Technical University-Kadoorie (PTUK), P.O. Box 7, Jaffa Street, Tulkarm, State of Palestine

## Abstract

Detection of food spoilage with simple and fast methods is an important issue in food security and safety. The present study is mainly aimed at identifying and quantifying four yeast species in white fresh soft cheese using an electronic nose (EN). The yeast species *Pichia anomala*, *Pichia kluyveri*, *Hanseniaspora uvarum*, and *Debaryomyces hansenii* were used. Six concentrations of each yeast species (100, 200, 400, 600, 800, and 1000 cells/g cheese) were inoculated in 100 g of fresh soft cheese and incubated for 48 h at 25°C. The EN was used to identify and quantify different yeast species in cheese samples. It was found that EN was able to discriminate between four yeast species using principal component analysis (PCA). Moreover, EN was able to quantify in good precision three (*Pichia anomala*, *Pichia kluyveri*, and *Debaryomyces hansenii*) of the four tested yeasts presented in cheese samples using partial least squares (PLS) models. It seems that EN is a reliable tool that can be used as a fast technique to identify and quantify cheese spoilage in the cheese industry.

## 1. Introduction

Fresh soft cheese is one of the perishable dairy products that is a preferred medium for microbial growth. Due to their lipolytic and proteolytic activities and ability to assimilate or ferment lactose and to assimilate organic acids, yeasts are found in raw milk and cheeses. Yeasts of the genera *Debaryomyces*, *Pichia*, *Geotrichum*, *Kluyveromyces Saccharomyces*, *Torulaspora*, *Trichosporon*, and *Yarrowia* were detected in white soft cheeses causing their spoilage [1–3]. The growth of yeasts in fresh white cheeses causes off-flavours, softening, gas production, discolouration, and swollen packages [4]. Contamination of white fresh cheese with yeasts will decrease their shelf life and affect their quality. On the other hand, the presence of yeast and *Yarrowia lipolytica* in some types of ripened cheeses is desirable as they contribute to the ripening process [5]. *Debaryomyces hansenii* was reported to promote the growth of *Brevibacterium linens* and increase the yellow colour intensity in Danish surface-ripened cheeses [6].

One of the main causes of economic losses for the food industry is microbial contamination. Furthermore, the growth of foodborne pathogens can lead to toxic food, which will cause severe diseases for the consumers. Yeasts are among the microorganisms that are known to cause food spoilage. The presence of yeasts in fresh cheeses will lead to off-flavour, discolouration, softening, and gas production. *Debaryomyces hansenii* and *Pichia anomala* were found among spoilage yeast isolated from Turkish fresh cheese [7]. Furthermore, *Hanseniaspora uvarum* and *Pichia kluyveri* have been isolated from yoghurt and fermented milk causing their spoilage [8]. Identification and quantification of yeast species in white fresh cheese rely on traditional microbial culture methods. Those methods are based on the isolation of yeasts from cheese samples by culturing them on culture media followed by characterization of physiological properties like growth requirements, assimilation, and fermentation. Further characterization and identification of yeast are carried out by molecular methods. For example, sequence analysis of the D1/D2 region of the 26S rRNA gene was used to identify yeast species in green coffee beans [9] and fresh white cheese [10]. Traditional molecular methods for the identification and quantification of microorganisms present in food products are time-consuming and high cost. For the food industry, reliable fast methods are needed to detect microbial contamination in food products.

An electronic nose (EN) is a sensor array that belongs to chemical sensors. EN mimics the olfaction system of the human. It is based on detecting volatile organic compounds (VOCs). It has been successfully used in several biological and agricultural applications [11, 12], especially in food spoilage [13–18]. Furthermore, it was used for the identification of several bacterial strains and fungi strains, since these microorganisms can produce VOCs during their metabolic activities. Mota et al. [17] reviewed the fungal species that were identified using different types of EN, due to its advantages.

The main goal of this research was to study the feasibility of the identification and quantification of four yeast species in white fresh cheese using EN. Six concentrations of *Pichia anomala* (PA), *Pichia kluyveri* (PK), *Debaryomyces hansenii* (DH), and *Hanseniaspora uvarum* (HU) were investigated. To our best knowledge, these species were not studied before using EN.

## 2. Materials and Methods

### 2.1. Yeast Species and Cheese Samples

Four species of yeast were used in the present study. They included *Debaryomyces hansenii*, *Pichia anomala*, *Pichia kluyveri*, and *Hanseniaspora uvarum*.

Fresh soft cheese was purchased from the local market. For each yeast species, 6 samples of 100 g of cheese were placed in sterile glass beakers.

### 2.2. Culture Media

The yeast culture medium Malt Yeast Glucose Peptone broth (MYGP) was prepared by dissolving 3 g of malt extract (Difco 0186-17), 3 g of yeast extract (Difco 0127-17), and 3 g of bactopeptone (Difco 0118-17) and 10 g D(+)-glucose monohydrate (Merck 8342) in 1 L distilled water. The pH of MYGP was adjusted to 5.6 by 1 M HCl or 1 M NaOH. Diluent saline peptone (SPO) was prepared by dissolving 8.5 g NaCl (Merck 6404), 0.3 g disodium hydrogen phosphate (Na_2_HPO_4_.12H_2_O; Merck 6579), and 1 g bactopeptone (Difco 0118-17) in 1 L distilled water and adjusted to pH 5.6 with the addition of 1 M HCl or 1 M NaOH. The two media were sterilized by autoclaving at 121°C for 15 min.

### 2.3. Yeast Inocula

Each yeast species was propagated in 25 ml of MYGP broth and incubated for 48 h at 25°C. Whereafter, yeast numbers were estimated under the microscope using a haemocytometer (Neubauer). From the number of each yeast cells estimated, six concentrations (100, 200, 400, 600, 800, and 1000 cells/g cheese) were adjusted by preparing cell suspensions in SPO. Each cheese sample (100 g) was inoculated with one of the six concentrations of each yeast species. The inoculated cheese samples were covered with a layer of parafilm and incubated at 25°C for 48 h to activate yeast cells. The experiment was conducted in triplicates for each concentration of yeast species. Negative control of cheese without yeast was used.

### 2.4. Electronic Nose (EN)

The EN device used in this research was a prototype. It consisted of eight metal-oxide semiconductors (MOSs) (Hanwei Electronics Co., Ltd., Zhengzhou, China). The specification of sensors can be found in Table 1. Each sample of cheese (i.e., 4 species with 5 concentrations (100, 200, 400, 600, 800, and 1000 cell/gram cheese)) was inserted inside a homemade box for about 5 minutes and measured in triplicates.

Table 1 is reproduced from Abu-Khalaf [11] (under the Creative Commons Attribution License/public domain).

### 2.5. Data Analysis

The Unscrambler (version 10.3, Camo Software AS, Oslo, Norway), which is a multivariate data analysis (MVDA) software, was used to reveal the relationship between the odour from cheese samples and the EN's signals.

Signals of EN for each sample were averaged and autoscaled. Principal component analysis (PCA) score plots were used to investigate the trend of the behaviour of measured samples. Partial least squares (PLS-1) models were used for quantification of different concentrations of four species (i.e., PLS-1: one model was created for each strain's concentration separately). Full cross-validation was used, due to the small number of samples [18, 21].

The evaluation of PLS-1 models was based on several factors, i.e., coefficient of correlation (*R*^2^), slope, and root mean square error (RMSE). Moreover, the ratio performance deviation (RPD) and relative error (RE) values were used to evaluate whether the PLS-1 models were accepted or rejected. RPD is defined as the ratio between the standard deviation of the response variable and RMSE.

A value less than 2.0 for RPD would indicate a poor model, while a value between 2.0 and 3.0 is considered an acceptable model, and a value greater than 3 shows an excellent prediction capability. For further details about evaluating models, the reader can refer to [19–22].

## 3. Results and Discussion

### 3.1. Electronic Nose (EN)

The maximum standard deviation and coefficient of variation (CV%) for the averages of all triplicates samples measured by EN were 22.5 mV and 3%, respectively. Three sensors (i.e., MQ-2, MQ-135, and MQ-138) were used for data analysis. These sensors gave the best classification and prediction results during data analysis trials for the four measured species samples.

### 3.2. Classification of Yeast Species

PCA score plot is shown in Figure 1. The first principal component (PC-1) explained 87% of the total variation, while the second principal component (PC-2) explained 11% of the data. Both PCs explained 98% of the total variation.

It can be seen that there is a clear classification between some species. *Pichia kluyveri* (PK) and *Pichia anomala* (PA) strains formed two clear groups as shown in Figure 1(a). However, the PK group showed less variation than the PA group. This might be explained by the headspace volatiles of those two yeasts. Masoud et al. [23] investigated the profiles of the volatiles produced by *P. anomala*, *P. kluyveri*, *H. uvarum*, and *D. hansenii*. It was found that *P. anomala* and *P. kluyveri* had very similar volatile profiles with variations in volatile concentrations. On the other hand, the volatile profile of *H. uvarum* was different from those of *P. anomala* and *P. kluyveri*, where some volatiles like isoamyl alcohol were not detected.

The other two species, i.e., *Debaryomyces hansenii (DH)* and *Hanseniaspora uvarum (HU)* overlapped each other, and no clear classification can be seen. This might also be due to the different selectivity and sensitivity of sensor array in EN for different volatile compounds secreted by different species. Different volatile profiles of those two species were reported [23].

Figure 1 also shows that EN was able to follow the concentration of PA. This can help in following the extent of spoilage and deterioration that can happen generally in food.

### 3.3. Prediction Models for Different Stains' Concentrations

Table 2 shows the results of partial least squares (PLS-1) models for quantification for each species with six concentrations. It can be noticed that the highest slope, *R*^2^, and RPD were for PA, DH, and PK strains. However, the lowest values were for HU strain.

RPD was used to determine if the model is accepted or not, depending on if its value is greater than 2. It was clear that all the models were accepted, except for the HU model. RPD values for PA, PK, and DH in the calibration set were 6.75, 5.05, and 7.49, respectively. RPD for HU was 1.58 (i.e., less than 2); consequently, its model was rejected.

The same trend can be seen in the validation set results. The RE for PK was the highest (i.e., 7.65%) in the calibration set, and the RE was the highest (i.e., 17.1%) for DH in the validation set models among the three accepted models.

It can be seen that three species were successfully modelled taking into consideration that their models have high *R*^2^, high slopes, low REs, and high RPDs. Nevertheless, there were differences between the calibration and validation parameters' values, which indicate the models can be considered as acceptable models. However, further investigation is needed for choosing different sensors for each species and not just using the best three common sensors for all species. Choosing three MOS for classification and prediction of the volatile compounds that are emitted by the four species may help in producing a quality control automatic monitoring system that can be used in the food storage room.

Related to a recent study carried by Masoud et al. [24], there was a contribution to model a concentration of one *D. hansenii* strain using EN [25]. The results in that contribution were that *R*^2^ and slope for the calibration set were both 0.97, while *R*^2^ and slope in the validation set were 0.95 and 0.99, respectively. Those results are a bit different from the results that we have got in the validation set in the current paper (i.e., *R*^2^ and slope are 0.83 and 1.04, respectively). This may be due to that the sensors chosen for building the PLS-1 models were different. This can also be attributed to growth differences between two tested strains of *D. hansenii*.

This research was an attempt to use EN as a sensor array technology for quality control of food spoilage. However, further research is needed to investigate more foods and different EN sensors that can help in future agricultural and biological applications.

## 4. Conclusions

The EN was able to discriminate between *P. anomala*, *P. kluyveri*, *H. uvarum*, and *D. hansenii* in fresh soft cheese. Furthermore, EN was able to quantify successfully three (i.e., *P. anomala*, *P. kluyveri*, and *D. hansenii*) of the four tested yeast species in fresh cheese. The present study demonstrated that EN is a fast and valid analytical equipment that can be used to identify and quantify yeast species when contaminating fresh soft cheeses. It has the potential to be used as an alarm system in food storage.

## Figures and Tables

**Figure 1:** Principal component analysis (PCA) score plot for measured contaminated cheese samples showing the concentration of four species using electronic nose (EN). *Pichia anomala* (PA), *Pichia kluyveri* (PK), *Debaryomyces hansenii* (DH), and *Hanseniaspora uvarum* (HU). Each name in the figure is followed by the concentration in cells/g.

**Table 1:** The characteristics of the eight metal-oxide semiconductor (MOS) sensors, which electronic nose (EN) is composed of.

Sensor name	Target gas sensitivity	Typical detection ranges (ppm)
MQ-2	General combustible gas	200–5000 liquefied petroleum gas (LPG) and propane, 300–5000 butane, 5000–20,000 methane, 300–5000 hydrogen (H_2_), 100–2000 alcohol
MQ-3	Alcohol vapour	10–300
MQ-4	Natural gas and methane	200–10,000 CH_4_, natural gas
MQ-5	Liquefied petroleum gas, natural gas, and coal gas	200–10,000 LPG, liquefied natural gas (LNG), natural gas, isobutane, propane, and town gas
MQ-6	LPG, propane	200–10,000 LPG, isobutane, propane, LNG
MQ-8	Hydrogen	100–10,000
MQ-135	Air quality control (NH_3_, benzene, alcohol, smoke)	10–10,000
MQ-138	Formaldehyde, benzene, aldehyde, ketone, and ester	10–1000 benzene, 1–1000 alcohol, 10–3000 NH_3_

**Table 2:** Results of partial least squares (PLS-1) models for four strains using electronic nose (as *X* matrix) and the concentration of each strain (as *Y* matrix) using three sensors (MQ-2, MQ-135, and MQ-138). The different parameters are shown in calibration and validation methods. Full cross-validation was used.

Parameters	Species names			
	*Pichia anomala* (PA)	*Pichia kluyveri* (PK)	*Debaryomyces hansenii (DH)*	*Hanseniaspora uvarum (HU)*
Calibration set				
*R*^2^	0.97	0.95	0.97	0.67
Slope	0.97	0.95	0.97	0.68
RMSE	50.96	67.64	46.17	181.2
RE (%)	5.56	7.65	5.20	20.13
Number of PCs used in the model	2	2	3	2
% of *X* explained	99	93	100	99
% of *Y* explained	98	96	98	79
RPD	6.75	5.05	7.49	1.58
Model performance	Acceptable	Acceptable	Acceptable	Rejected
Validation set				
*R*^2^	0.88	0.86	0.83	0.51
Slope	0.80	0.76	1.04	0.52
RMSE	128.87	144.76	15.89	266.21
RE (%)	14.20	16.18	17.12	29.57
Number of PCs used in the model	2	2	3	2
% of *X* explained	99	93	100	99
% of *Y* explained	98	96	98	79
RPD	2.36	2.04	2.63	1.31
Model performance	Acceptable	Acceptable	Acceptable	Rejected

*R* ^2^: correlation coefficient; RMSE: root mean square error; RE: relative error (i.e., RE = RMSE/range); PCs: principal components; RPD: ratio performance deviation (RPD = standard deviation of the *Y* − predicted/RMSE).

## Data Availability

Data is available on request.
